The article "Identification and Validation of Ferroptosis-Related Genes in Sevoflurane-Induced Hippocampal Neurotoxicity" was published in 2022. Journal: Oxid Med Cell Longev.

# Identification and Validation of Ferroptosis-Related Genes in Sevoflurane-Induced Hippocampal Neurotoxicity

**DOI:** 10.1155/2022/4435161

**Published:** 2022-10-04

**Authors:** Mengrong Miao, Yangyang Wang, Shuang Zeng, Yaqian Han, Ruilou Zhu, Pengfei Yu, Yitian Yang, Ningning Fu, Ningning Li, Mingyang Sun, Jiaqiang Zhang

**Affiliations:** ^1^Department of Anesthesiology and Perioperative Medicine, People's Hospital of Zhengzhou University, Henan Provincial People's Hospital, People's Hospital of Henan University, Zhengzhou, 450003 Henan Province, China; ^2^Department of Hepatobiliary and Pancreatic Surgery, People's Hospital of Zhengzhou University, Henan Provincial People's Hospital, People's Hospital of Henan University, Zhengzhou, 450003 Henan Province, China

## Abstract

**Background:**

Sevoflurane is one of the most popular inhalational anesthetics during perioperative period but presenting neurotoxicity among pediatric and aged populations. Recent experiments in vivo and in vitro have indicated that ferroptosis may contribute to the neurotoxicity of sevoflurane anesthesia. However, the exact mechanism is still unclear.

**Methods:**

In current study, we explored the differential expressed genes (DEGs) in HT-22 mouse hippocampal neuronal cells after sevoflurane anesthesia using RNA-seq. Differential expressed ferroptosis-related genes (DEFRGs) were screened and analyzed by Gene Ontology (GO) and pathway enrichment analysis. Protein-to-protein interaction (PPI) network was constructed by the Search Tool for the Retrieval of Interacting Genes (STRING). Significant modules and the hub genes were identified by using Cytoscape. The Connectivity Map (cMAP) was used for screening drug candidates targeting the identified DEFRGs. Potential TF-gene network and drug-gene pairs were established towards the hub genes. In final, we validated these results in experiments.

**Results:**

A total of 37 ferroptosis-related genes (18 upregulated and 19 downregulated) after sevoflurane exposure in hippocampal neuronal cells were finally identified. These differentially expressed genes were mainly involved into the biological processes of cellular response to oxidative stress. Pathway analysis indicated that these genes were involved in ferroptosis, mTOR signaling pathway, and longevity-regulating pathway. PPI network was constructed. 10 hub genes including Prkaa2, Chac1, Arntl, Tfrc, Slc7a11, Atf4, Mgst1, Lpin1, Atf3, and Sesn2 were found. Top 10 drug candidates, gene-drug networks, and TFs targeting these genes were finally identified. These results were validated in experiments.

**Conclusion:**

Our results suggested that ferroptosis-related genes play roles in sevoflurane anesthesia-related hippocampal neuron injury and offered the hub genes and potential therapeutic agents for investigating and treatment of this neurotoxicity after sevoflurane exposure. Finally, therapeutic effect of these drug candidates and function of potential ferroptosis targets should be further investigated for treatment and clarifying mechanisms of sevoflurane anesthesia-induced neuron injury in future research.

## 1. Introduction

Millions of patients received surgery and anesthesia every year in the world. As one of the most popular inhalational anesthetics during general anesthesia, sevoflurane acted rapidly with high acceptance but was associated with perioperative neurocognitive disorders (PND) [1–3]. The wide application of sevoflurane during general anesthesia makes its safety a major health concern. Hence, precise strategy against sevoflurane-induced neurotoxicity and learning and memory impairment are urgently needed. However, to date, the mechanisms of sevoflurane-induced neuronal injury was not fully understood, which poses a barrier to the treatment of its neurotoxicity.

Different from any existing types of cell death such as apoptosis, autophagy, pyroptosis, or necrosis, ferroptosis presents as a new form of programmed cell death characterized by excessive accumulation of iron and lipid peroxidation [4]. Ferroptosis in neuronal cells was associated with many diseases in CNS, such as Alzheimer's disease [5, 6], epilepsy [7], and neonatal brain injury [8]. Recently, several studies focused on sevoflurane anesthesia-induced cognitive impairment also found the involvement of ferroptosis in neuronal cells [9–12]. In 2020, Wu et al. reported that sevoflurane anesthesia contributed iron overload and ferroptosis in hippocampal neurons, which may be activated by NMDAR-RASD1 signaling via DMT1 action [9]. Cheng et al. found sevoflurane-induced ferroptotic neuronal death in SH-SY5Y cells, which was associated with the involvement of ACSL4 [10]. In addition, ferroptosis modulated sevoflurane-induced cognitive impairment through interaction between Mind bomb-2 (Mib2) and glutathione peroxidase 4 (Gpx4) [11]. All these studies indicated that targeting ferroptosis is supposed to be an effective strategy for treating sevoflurane-induced brain injury.

In this study, with the help of bioinformatics, we investigated the differential expressed genes (DEGs) in HT22 hippocampal neuronal cells after sevoflurane exposure through RNA-seq. Ferroptosis-related genes (FRGs) and pathways that may play important role in sevoflurane anesthesia-induced neurotoxicity were identified. Potential therapeutic agents targeting to differentially expressed ferroptosis-related genes (DEFRGs) and their hub genes were also explored and validated.

## 2. Materials and Methods

### 2.1. Cell Processing and RNA Sequencing

In current study, the mouse HT22 hippocampal neuronal cells employed were purchased from CHI Scientific (Shanghai, China). The hippocampal neuronal cells were maintained in DMEM medium containing 10% fetal bovine serum (FBS) and 1% penicillin–streptomycin (PS) at 37°C in 5% CO2 cell incubator. Cells were randomly divided into a control group and a sevoflurane group. In the sevoflurane group, the HT22 cells were put in a gas-tight chamber and were exposed to 4% sevoflurane for 24 hours. The cells in the control group were put outside the chamber but in the same incubator during the process. After treatment, total RNA of HT22 cells in each group was extracted by using the TRIzol reagent. The cDNA was obtained from 1 *μ*g of total RNA by reverse transcriptase. RNA sequencing was performed on DNBSEQ platform by BGI genomics (Beijing, China).

### 2.2. Identification of Differentially Expressed Genes (DEGs)

Expression of 18559 genes in HT22 cells was compared between the control group and the sevoflurane group. Deseq2 package (1.34.0) was used to identify DEGs after sevoflurane exposure. Genes with *p* value <0.05 and a |log2FoldChange| >1 were defined as DEGs. DEGs were visualized through heatmap which is generated by pheatmap package (1.0.12).

### 2.3. Identification of DEFRGs

Ferroptosis-related genes were extracted from GeneCards (Version 5.9, https://www.Genecards.org/). An online bioinformatic tool (http://bioinformatics.psb.ugent.be/webtools/Venn/) was used to draw Venn diagrams between tested 18559 genes and 442 FRGs in GeneCards and then overlapped with sevoflurane-induced DEGs. Subsequently, overlapped DEGs were included into subsequent analyses.

### 2.4. Gene Ontology and Pathway Enrichment Analyses

Enrichment analysis of Gene Ontology (GO) was performed to illustrate the function of significant DEGs in biological process by using the clusterProfiler package (4.2.2). The Kyoto Encyclopedia of Genes and Genomes (KEGG) pathway analysis of significant DEGs was also investigated by using the clusterProfiler package (4.2.2) and the ggplot2 package (3.3.6) in R studio.

### 2.5. Construction of Protein-Protein Interaction (PPI) Network and Module Analysis

To identify potential interaction relationship between target genes-encoded proteins, a PPI network was constructed by using online database STRING (version 11.5, https://cn.string-db.org/). Required interaction score of 0.15 was set as a threshold value. After that, the results of STRING were imported into the Cytoscape software (3.9.0) to build the PPI network of the whole FRGs. Then the Molecular Complex Detection (MCODE) plug-in was used to screen significant PPI network modules. We set the criteria as the following: degree cut − off = 2, node score cut − off = 0.2, max depth = 100, and *k* − score = 2. After that, the GO and KEGG analysis of the involved modular genes were conducted by using the clusterProfiler package (4.2.2) and the ggplot2 package (3.3.6) in R studio.

### 2.6. Selection and Analysis of the Hub Genes

CytoHubba plug-in of Cytoscape was used to identify the hub genes. Eight different algorithms (MCC, DMNC, MNC, degree, closeness, radiality, stress, and EPC) were calculated for screening and selecting reliable hub genes. Then a coexpression network of the hub genes and their coexpressed genes was established based on GeneMANIA (http://www. http://genemania.org/) [13].

### 2.7. Screening of Potential Therapeutic Candidates

To screen for therapeutic agents targeting to FRGs analyzed from PPI network, the Connectivity Map (cMAP) database (https://clue.io/query) was utilized. The cMAP is an online database cataloging gene expression profiling from cultured cell lines treated by various small molecule compounds. By comparing the similarities of FRGs and drug-induced gene expression profiles, the cMAP could predict potential drug candidates through generating a connectivity score ranged from -100 to 100. In addition, a drug–hub gene interaction network for finding therapeutic drugs towards to the hub genes was also established with DGIdb database (http://dgidb.genome.wustl.edu/) and visualized by Cytoscape.

### 2.8. Transcription Factors (TFs) Prediction

We submitted the hub genes to ChIP-X Enrichment Analysis 3 (ChEA3) platform for TF prediction revealed by transcription factor enrichment analysis (https://maayanlab.cloud/chea3/#top) [14]. Predicted hub gene-associated TFs were ranked by mean rank score.

### 2.9. Quantitative Real-Time PCR (qPCR)

The primers of target genes were obtained from the PrimerBank (https://pga.mgh.harvard.edu/primerbank/index.html). Total RNA was reversed into cDNA using the HiScript® III RT SuperMix (Cat. R223-01, Vazyme, China). Real-time PCR assays were performed using the AceQ®qPCR SYBR Green Master Mix Kit (Cat. Q711-02, Vazyme, China). The primer sequences of these genes are summarized in Table 1. The relative levels of target genes were quantified using 2−*ΔΔ*Ct method and were normalized to *β*-actin.

### 2.10. Measurements of Cell Viability and Glutathione (GSH) Levels

Cell Counting Kit-8 (CCK8, Cat. C0037, Beyotime, China) was used to evaluate cell viability after sevoflurane exposure according to the manufacturer's instructions. C cellular GSH levels were detected by a GSH Assay Kit (Cat. S0058, Beyotime, China).

### 2.11. Western Blotting

After sevoflurane exposure, HT22 cells were lysed in precooled RIPA lysis buffer (Cat. R0020, SolelyBio, China) with protease inhibitor (Cat. M5293, AbMole, USA). We quantified the protein using a BCA Protein Quantitation Kit (Cat. PC0020, SolelyBio, China). The equal protein in each group was separated in 10% SDS PAGE (Cat. LK303, Epizyme, China) and transferred into PVDF membrane (Cat. ISEQ00010, Millipore, USA). The primary antibodies used in this study were anti-Slc7a11 (Cat. ab175186, Abcam, dilution 1 : 1000), anti-Gpx4 (Cat. AB_2838663, Affinity, dilution 1 : 1000), and anti-GAPDH (Cat. 60004-1-Ig, Proteintech, dilution 1 : 1000). Super ECL detection reagent (Cat. SQ101, Epizyme, China) was used for visualizing the protein bands in PVDF membrane. ImageJ 1.53 software was used for quantification of the protein bands.

### 2.12. Statistical Analysis

Statistical analyses were performed by GraphPad Prism 8 (GraphPad Software, Inc.). Normality of results was checked by the Shapiro–Wilk test. Data were presented as mean ± SD and calculated with unpaired two-tailed Student's *t*-test when they were normally distributed. Otherwise, data were presented as median and differences and calculated with the Mann–Whitney *U* test. Two-sided *p* < 0.05 was considered statistically significant.

## 3. Results

### 3.1. Identification of DEGs and DEFRGs

Flowchart of the present study is shown in Figure 1. In this study, we obtained 1459 DEGs in HT22 hippocampal neuronal cells after sevoflurane exposure (Figure 2(a)). Among 18559 tested genes in HT22 cells, 378 genes were associated with ferroptosis (Figure 2(b)). Venn diagram of 378 FRGs and sevoflurane-induced 1459 DEGs indicated 37 DEFRGs after sevoflurane exposure (Figure 2(c), hypergeometric distribution test showed *p* value =0.03). Expression levels of 37 DEFRGs were presented in heatmap (Figure 2(d)).

### 3.2. GO and KEGG Pathway Enrichment Analysis of DEFRGs

GO and KEGG pathway enrichment analysis were performed to identify 37 DEFRGs that involved biological functions and pathways. GO analysis indicated that these genes were mainly involved in response to oxidative stress, cellular response to oxidative stress, cellular response to chemical stress, glucose metabolic process, cellular response to extracellular stimulus, regulation of transcription from RNA polymerase II-promoter in response to stress, and regulation of DNA-templated transcription in response to stress (Figure 3(b)). KEGG pathway analysis demonstrated that DEFRGs after sevoflurane exposure were main involved in ferroptosis, mTOR signaling pathway, longevity regulating pathway, circadian rhythm, and alcoholic liver disease (Figure 3(c)). Among which, 19 upregulated FRGs were mainly involved in alcoholic liver disease, mTOR signaling pathway, and glycerolipid metabolism, while 18 downregulated FRGs were mainly involved in ferroptosis, central carbon metabolism in cancer, and longevity regulating pathway (Figure 3(d)).

### 3.3. PPI Network Construction and Module Analysis

PPI network of FRGs involving 37 nodes and 128 edges was constructed by STRING and was visualized by Cytoscape (Figure 3(a)). Three significant modules were found by MCODE plug-in of Cytoscape (Figure 4(a)). GO analysis of modular genes indicated that these genes are associated with regulation of cellular amide metabolic process, regulation of small molecule metabolic process, and response to oxidative stress (Figure 4(b)). KEGG pathway analysis demonstrated that these genes were mainly involved in circadian rhythm, ferroptosis, mTOR signaling pathway, phagosome, central carbon metabolism in cancer, and longevity regulating pathway (Figure 4(c)). KEGG pathway enrichment of up- and downregulated modules genes is separately analyzed and shown in Figure 4(d).

### 3.4. Selection and Analysis of the Hub Genes

The top 20 hub genes were calculated by using CytoHubba plug-in through 8 different algorithms (MCC, DMNC, MNC, degree, closeness, radiality, stress, and EPC). Upset diagram of results of these algorithms (Table 2) revealed that 10 common hub genes involving Prkaa2, Chac1, Arntl, Tfrc, Slc7a11, Atf4, Mgst1, Lpin1, Atf3, and Sesn2 were found (Figure 5(a)). Full names and descriptions of these hub genes are summarized in Table 3. The coexpression network and associated functions of these genes was established via GeneMANIA database. These genes showed the complex PPI network with the coexpression of 96.17%, prediction of 1.83%, colocalization of 0.84%, and shared protein domains of 0.14% (Figure 5(b)). GO analysis showed that these hub genes were related to cellular response to oxidative stress, cellular response to chemical stress, and response to oxidative stress (Figure 5(c)). KEGG pathway analysis indicated that they were mainly involved in longevity regulating pathway, circadian rhythm, mTOR signaling pathway, and ferroptosis (Figure 5(d)).

### 3.5. Prediction and Expression of TFs

Given the critical role of TFs in regulation of gene transcription and expression, a list of the hub genes was submitted to ChEA3 platform for transcription factor enrichment analysis. TFs regulatory network of top10 TFs and the hub genes is shown in Figure 6(a). The expression of top10 TFs is presented in Figure 6(b). Among them, Zbed6 was highly expressed, while Egr1 was lowly expressed in mouse hippocampal neuronal cells after sevoflurane exposure (*p* value <0.05 and |log2FoldChange| >1).

### 3.6. Drug Candidates for DEFRGs and the Hub Genes

The Connectivity Map (cMAP) collected the gene-expression signatures in response to small molecule compounds. To find drug candidates for targeting DEFRGs, cMAP was queried for potential compounds (at least inputted 10 up and down genes are needed for this database). A list of top10 ranked small molecular compounds is summarized in Figure 7(a). In addition, to minimize the treatment scope, drug targeting 10 hub genes was predicted. After prediction, gene-drug networks involving 4 hub genes and 9 drugs could be established via DGIdb database (Figure 7(b)).

### 3.7. Validation of Genes Expression in Hippocampal Neuronal Cells after Sevoflurane Exposure

Figure 8 reveals the ferroptosis of hippocampal neuronal cells after sevoflurane treatment. Sevoflurane exposure increased the mRNA expression of Ftl1 and Ptgs2 and decreased GSH and cell viability in HT22 cells (Figures 8(a)–8(g)). The expression of Slc7a11 and Gpx4 protein was also significantly downregulated by sevoflurane (Figures 8(d)–8(g)). The expression of Prkaa2, Mgst1 Lpin1, and Tfrc were significantly increased after sevoflurane treatment (*p* < 0.05) (Figures 8(h)–8(k)). Chac1, Arntl, Slc7a11, Atf3, and Sesn2 were significantly decreased after sevoflurane exposure (*p* < 0.05), while the expression of Atf4 were not changed after sevoflurane exposure (Figures 8(l)–8(q)). We also validated the expression of predicted significant TFs (Egr1 and Zbed6). qPCR verified the high expression of Zbed6 in sevoflurane-anesthetized HT22 cells.

## 4. Discussion

Sevoflurane induced neurotoxicity through many complex processes. However, the exact mechanisms were not fully understood. In the current study, we investigated DEFRGs after sevoflurane exposure for providing a new insight into underlying mechanism of sevoflurane-induced neuronal injury in transcriptional level. After overlapping of tested FRGs and sevoflurane-induced DEGs, 37 DEFRGs were found. PPI and enrichment analysis of these genes were performed. GO analysis showed that these DEFRGs were mainly involved in oxidative stress, while KEGG analysis demonstrated that these genes were mainly involved in ferroptosis, mTOR signaling pathway, and longevity regulating pathway. In addition, we found three significant modules using MCODE plug-in of Cytoscape; in GO and KEGG analysis of module genes, oxidative stress, ferroptosis, mTOR signaling pathway, and longevity regulating pathway were also enriched. These above results provided new reference for treatment of sevoflurane's neurotoxicity. Furthermore, we submitted the DEFRGs in cMAP database to predict potential compounds for treatment of sevoflurane-induced neuronal injury. Top 10 of them were ABT-751, practolol, KUC103420N, pioglitazone, GSK-3-inhibitor-II, VU-0365114-2, cycloheximide, avrainvillamide-analog-1, phensuximide, and VX-222. Their therapeutic role in sevoflurane-induced neuronal injury is worth exploring.

Of the 37 DEFRGs, 10 genes including Prkaa2, Chac1, Arntl, Tfrc, Slc7a11, Atf4, Mgst1, Lpin1, Atf3, and Sesn2 were identified as the hub genes via overlapping of 8 algorithms of CytoHubba. Prkaa2, protein kinase AMP-activated catalytic subunit alpha 2, is a catalytic subunit of the AMP-activated protein kinase (AMPK) which was an important energy-sensing enzyme that monitors cellular energy status. Prkaa2 can mediate autophagy through targeting to key autophagy-related proteins such as ULK1 or through regulating the activity of mTOR [15]. Chac1 encodes a member of the gamma-glutamylcyclotransferase family of proteins, which is involved in neuronal differentiation by deglycination of the Notch receptor [16]. Arntl is a basic helix-loop-helix protein that forms a heterodimer with CLOCK. The selective degradation of Arntl by autophagy facilitates ferroptosis induction [17]. Slc7a11, solute carrier family 7 member 11, the subunits of System Xc-, is responsible for transportation of cysteine and glutamate [18]. Inhibition of the expression of Slc7a11 could affect the activity of Gpx4, induce decline of GSH and accumulation of lipid ROS, and finally lead to ferroptosis [19]. Atf4, activating transcription factor 4, is a member of DNA-binding proteins that includes the AP-1 family of transcription factors, cAMP-response element binding proteins (CREBs) and CREB-like proteins [20–23]. Atf4 presented a protective role in oxidative stress and endoplasmic reticulum stress [24, 25]. Atf3, activating transcription factor 3, also encoded a member of the mammalian activation transcription factor/cAMP responsive element-binding (CREB) protein family of transcription factors [26]. It is involved in the complex process of cellular stress response. A latest study indicated that ATF3 was involved in neuronal differentiation and development of neuronal networks in opossum postnatal cortical cultures [27]. Sesn2, sestrin2, is a highly conserved antioxidative protein which was activated in various stress [28]. It was reported that Sesn2 served as a protective gene against sepsis-induced ferroptosis and iron overload and ferroptosis-induced liver injury [29, 30]. Coexpression network established by GeneMANIA database showed that these hub genes and their coexpression genes were mainly enriched in endoplasmic reticulum stress.

Furthermore, TFs may regulate that these genes were investigated. In top10 TFs predicted by mean rank scores of ChEA3, Egr1 and Zbed6 were differently expressed in mouse hippocampal neuronal cells after sevoflurane exposure (log2FoldChange of -2.30 and 1.77). Egr1, early growth response 1, participated in the regulation of synaptic plasticity and neuronal activity [31, 32]. The Egr-1 regulates ferroptosis in acute myocardial infarction through miR-15a-5p/GPX4 axis [33], while GPX4 regulated mitochondria-mediated apoptosis through regulation of Egr1 in TNBC cells [34]. In CNS, Egr1 mRNA expression level was significantly decreased in cognitive dysfunction model of T2DM mice [35]. Zbed6, zinc finger BED domain-containing protein 6, established a role in regulating IGF2 mRNA expression and insulin production, maintaining beta cell area, and reducing excess mitochondrial activation [36–38].

In addition, to minimize the treatment scope, we investigated potential drug targeting to these hub genes separately in DGIdb database. 4 of 10 genes (Slc7a11, Prkaa2, Lpin1, and Atf3) could be predicted for drug candidates and could generate drug-gene networks.

We verified the occurrence of ferroptosis in hippocampal neuronal cells after sevoflurane treatment. Also, the expression of 10 hub genes and 2 significant TFs were validated by qPCR, and their changes after sevoflurane exposure were mostly consistent with RNA-seq.

Except for ferroptosis, the participation of autophagy in sevoflurane-induced hippocampal neuronal injury was verified in recent years [39]. Upregulation of autophagy marker LC3II/I and p62 after sevoflurane treatment were observed in hippocampus of neonatal or aged rats/mouse [40–42]. In a well-performed study, oxygen glucose deprivation and reoxygenation (OGD/R) of HT22 cells decreased the level of autophagy marker such as Lc3b, P62, and Pink1, Parkin, while sevoflurane postcondition (SP) improved the suppression of these genes and mitochondria dysfunction through Sirt1 [43]. Interestingly, autophagy-dependent ferroptosis proved a critical role in hippocampal neuronal injury recently [44–46]. In the current investigation on FRGs, autophagy was enriched in KEGG pathway analysis of the modular genes (Figure 4(c)). And in 10 hub DEFRGs, Prkaa2 [15], Arntl [17], Sesn2 [47], and Lamp2 [48] reported the involvement in autophagy, which may indicate a link between autophagy and ferroptosis in sevoflurane-induced hippocampal neuronal injury.

The current study has several limitations. First, we identified our finding in cell experiments, and further investigation will be confirmed in animal experiments. Second, the prediction results of drug candidates were not validated. We will confirm these finding in our further experiments.

## 5. Conclusion

In summary, this study identified DEFRGs after sevoflurane exposure and TFs, potential therapeutic candidates towards these genes, which may provide new clues for further studies on sevoflurane-induced neurotoxicity. Drug candidates and potential ferroptosis targets revealed by the current study should be further investigated for treatment and elucidating mechanisms of sevoflurane anesthesia-induced neurotoxicity in the subsequent studies.

## Figures and Tables

**Figure 1:** Flowchart of the present study. DEGs: differentially expressed genes; FRGs: ferroptosis-related genes; DEFRGs: differential expressed ferroptosis-related genes; cMAP: Connectivity Map; PPI: protein-protein interaction; GO: gene ontology; KEGG: Kyoto Encyclopedia of Genes and Genomes; MCODE: the Molecular Complex Detection; qPCR: quantitative real-time PCR; TF: transcription factor; ChEA3: ChIP-X Enrichment Analysis 3.

**Figure 2:** Identification of DEGs and DEFRGs after sevoflurane exposure. (a) Heatmap of DEGs after sevoflurane exposure; (b) Venn diagram of all detected genes and FRGs; (c) Venn diagram of sevoflurane-induced DEGs and detected FRGs; (d) heatmap of 37 DEFRGs.

**Figure 3:** PPI network and enrichment analysis of DEFRGs. (a) PPI network of DEFRGs; (b) GO enrichment analysis of the DEFRGs; (c) Cnetplot of KEGG pathway analysis of the DEFRGs; (d) The separative KEGG analysis for upregulated and downregulated DEFRGs.

**Figure 4:** The important gene modules and enrichment analysis of the modular genes. (a) Three significant modules filtered by MCODE; (b) GO enrichment analysis of the modular genes; (c) Cnetplot of KEGG pathway analysis of the modular genes; (d) The separative KEGG analysis for upregulated and downregulated modular genes.

**Figure 5:** Upset diagram, coexpression network, and enrichment analysis of the hub genes. (a) 10 overlapping hug genes calculated by 8 algorithms of CytoHubba; (b) coexpression network of the hub genes was established via GeneMANIA; (c) GO enrichment analysis of the hub genes; (d) KEGG pathway analysis of the hub genes.

**Figure 6:** Prediction and expression of TFs targeting the hub genes. (a) Interaction network of top10 TFs and the hub genes; (b) the heatmap of the expression of the top10 TFs revealed by RNA-seq (red arrows, significantly upregulated TF; blue arrows, significantly downregulated TF).

**Figure 7:** Drug candidates for ferroptosis-related DEGs and the hub genes. (a) Top 10 small molecular compounds for DEFRGs identified by cMAP database; (b) the drug–hub gene interaction network established by DGIdb database.

**Figure 8:** Validation of genes expression after sevoflurane anesthesia in hippocampal neuronal cells. (a) mRNA expression of Ftl1; (b) GSH content in HT-22 cells; (c) cell viability; (d–f) the expression of Slc7a11 and Gpx4 in HT22 cells; (g–s) mRNA expression of hub genes and significant TFs.

**Table 1:** The primer sequences of qPCR.

Gene	Forward primer (5′ to 3′)	Reverse primer (5′ to 3′)
Prkaa2	CAGGCCATAAAGTGGCAGTTA	AAAAGTCTGTCGGAGTGCTGA
Chac1	CTGTGGATTTTCGGGTACGG	CCCCTATGGAAGGTGTCTCC
Arntl	TCAAGACGACATAGGACACCT	GGACATTGGCTAAAACAACAGTG
Tfrc	GTTTCTGCCAGCCCCTTATTAT	GCAAGGAAAGGATATGCAGCA
Slc7a11	GGCACCGTCATCGGATCAG	CTCCACAGGCAGACCAGAAAA
Atf4	GTTTAGAGCTAGGCAGTGAAG	CCTTTACACATGGAGGGATTAG
Mgst1	CTCAGGCAGCTCATGGACAAT	GTTATCCTCTGGAATGCGGTC
Lpin1	CTCCGCTCCCGAGAGAAAG	TCATGTGCAAATCCACGGACT
Atf3	GAGGATTTTGCTAACCTGACACC	TTGACGGTAACTGACTCCAGC
Sesn2	AGCAGAGCTGGTTTAGTGAACCG	GACAAACCACAACTAGAATGC
Egr1	ACCCTATGAGCACCTGACCAC	TATAGGTGATGGGAGGCAACC
Zbed6	CAAGACATCTGCAGTTTGGAATTT	TGTCGTTGAAGTGTTGAAGTTCCTA
*β*-Actin	GGCTGTATTCCCCTCCATCG	CCAGTTGGTAACAATGCCATGT

**Table 2:** The top 20 hub genes indicated by CytoHubba.

MCC	DMNC	MNC	Degree	Closeness	Radiality	Stress	EPC
Myc	Etv4	Myc	Myc	Myc	Myc	Myc	Myc
Sesn2	Bach1	Snca	Chac1	Tigar	Snca	Dhx9	Chac1
Atf4	Slc7a11	Atf3	Snca	Lpin1	Sesn2	Tigar	Lpin1
Atf3	Lamp2	Sesn2	Lpin1	Mgst1	Atf3	Hnrnpm	Tigar
Slc7a11	Atf4	Atf4	Tigar	Snca	Ksr2	Lpin1	Sesn2
Snca	Foxc1	Ksr2	Sesn2	Chac1	Atf4	Mgst1	Snca
Chac1	Tigar	Tfrc	Atf4	Sesn2	Tfrc	Snca	Mgst1
Lpin1	Atf3	Lpin1	Tfrc	Atf3	Vim	Chac1	Atf4
Ksr2	Sesn2	Arntl	Eno2	Atf4	Lpin1	Atf3	Atf3
Bach1	Chac1	Prkaa2	Mgst1	Tfrc	Arntl	Eno2	Tfrc
Tfrc	Pfn2	Slc7a11	Atf3	Eno2	Mgst1	Tfrc	Prkaa2
Prkaa22	Lpin2	Mgst1	Prkaa2	Prkaa2	Slc7a11	Atf4	Eno2
Tubb4a	Prkaa2	Vim	Siah2	Dhx9	Lamp2	Sesn2	Slc7a11
Arntl	Ksr2	Eno2	Dhx9	Siah2	Prkaa2	Siah2	Siah2
Vim	Lpin1	Tubb4a	Slc7a11	Lamp2	Eno2	Prkaa2	Lamp2
Lamp2	Vim	Chac1	Hnrnpm	Etv4	Tubb4a	Etv4	Dhx9
Mgst1	Tubb4a	Lamp2	Lamp2	Arntl	Chac1	Lpin2	Etv4
Eno2	Arntl	Hnrnpm	Etv4	Slc7a11	Tigar	Arntl	Arntl
Foxc1	Tfrc	Bach1	Lpin2	Lpin2	Hnrnpm	Rbm10	Lpin2
Tigar	Mgst1	Foxc1	Arntl	Hnrnpm	Nolc1	Slc7a11	Vim

**Table 3:** Summary of 10 hub genes.

No	Gene symbol	Full name	Function
1	Prkaa2	Protein kinase AMP-activated catalytic subunit alpha 2	Prkaa2 is a catalytic subunit of the AMP-activated protein kinase (AMPK). AMPK is an important energy-sensing enzyme that monitors cellular energy status
2	Chac1	Chac glutathione-specific gamma-glutamylcyclotransferase 1	This gene encodes a member of the gamma-glutamylcyclotransferase family of proteins. Chac1 is involved in neuronal differentiation by deglycination of the Notch receptor
3	Arntl	Aryl hydrocarbon receptor nuclear translocator like	Arntl is a basic helix-loop-helix protein that forms a heterodimer with CLOCK. This heterodimer binds E-box enhancer elements upstream of period (PER1, PER2, PER3) and cryptochrome (CRY1, CRY2) genes and activates transcription of these genes
4	Tfrc	Transferrin receptor	Tfrc encodes a cell surface receptor necessary for cellular iron uptake by the process of receptor-mediated endocytosis. This receptor is required for erythropoiesis and neurologic development
5	Slc7a11	Solute carrier family 7 member 11	Slc7a11 is a member of a heteromeric, sodium-independent, anionic amino acid transport system. It is responsible for the transportation of cysteine and glutamate
6	Atf4	Activating transcription factor 4	Atf4 belongs to a family of DNA-binding proteins that includes the AP-1 family of transcription factors, cAMP-response element binding proteins (CREBs), and CREB-like proteins
7	Mgst1	Microsomal glutathione S-transferase 1	This gene encodes a protein that catalyzes the conjugation of glutathione to electrophiles and the reduction of lipid hydroperoxides
8	Lpin1	Lipin 1	Lpin1 encodes a magnesium-ion-dependent phosphatidic acid phosphohydrolase enzyme that catalyzes the penultimate step in triglyceride synthesis
9	Atf3	Activating transcription factor 3	Atf3 encodes a member of the mammalian activation transcription factor/CREB protein family of transcription factors. It is involved in the complex process of cellular stress response
10	Sesn2	Sestrin2	Sesn2 is a member of the sestrin family of PA26-related proteins. It may be involved in the regulation of cell growth and survival, cellular response to different stress conditions

## Data Availability

The data used to support the findings of this study are included within the article.
